The article "Correlation Evaluation of Pilots' Situation Awareness in Bridge Simulations via Eye-Tracking Technology" was published in 2021. Journal: Comput Intell Neurosci.

# Correlation Evaluation of Pilots' Situation Awareness in Bridge Simulations via Eye-Tracking Technology

**DOI:** 10.1155/2021/7122437

**Published:** 2021-12-03

**Authors:** Shaoqi Jiang, Weijiong Chen, Yutao Kang

**Affiliations:** College of Ocean Science and Engineering, Shanghai Maritime University, Shanghai, China

## Abstract

To maintain situation awareness (SA) when exposed to emergencies during pilotage, a pilot needs to selectively allocate attentional resources to perceive critical status information about ships and environments. Although it is important to continuously monitor a pilot's SA, its relationship with attention is still not fully understood in ship pilotage. This study performs bridge simulation experiments that include vessel departure, navigation in the fairway, encounters, poor visibility, and anchoring scenes with 13 pilots (mean = 11.3 and standard deviation = 1.4 of experience). Individuals were divided into two SA group levels based on the Situation Awareness Rating Technology (SART-2) score (mean = 20.13 and standard deviation = 5.83) after the experiments. The visual patterns using different SA groups were examined using heat maps and scan paths based on pilots' fixations and saccade data. The preliminary visual analyses of the heat maps and scan paths indicate that the pilots' attentional distribution is modulated by the SA level. That is, the most concerning areas of interest (AOIs) for pilots in the high and low SA groups are outside the window (AOI-2) and electronic charts (AOI-1), respectively. Subsequently, permutation simulations were utilized to identify statistical differences between the pilots' eye-tracking metrics and SA. The results of the statistical analyses show that the fixation and saccade metrics are affected by the SA level in different AOIs across the five scenes, which confirms the findings of previous studies. In encounter scenes, the pilots' SA level is correlated with the fixation and saccade metrics: fixation count (*p* = 0.034 < 0.05 in AOI-1 and *p* = 0.032 < 0.05 in AOI-2), fixation duration (*p* = 0.043 < 0.05 in AOI-1 and *p* = 0.014 < 0.05 in AOI-2), and saccade count (*p* = 0.086 < 0.1 in AOI-1 and *p* = 0.054 < 0.1 in AOI-2). This was determined by the fixation count (*p* = 0.024 < 0.05 in AOI-1 and *p* = 0.034 < 0.05 in AOI-2), fixation duration (*p* = 0.036 < 0.05 in AOI-1 and *p* = 0.047 < 0.05 in AOI-2), and saccade duration (*p* = 0.05 ≤ 0.05 in AOI-1 and *p* = 0.042 < 0.05 in AOI-2) in poor-visibility scenes. In the remaining scenes, the SA could not be measured using eye movements alone. This study lays a foundation for the cognitive mechanism recognition of pilots based on SA via eye-tracking technology, which provides a reference to establish cognitive competency standards in preliminary pilot screenings.

The article "Correlation Evaluation of Pilots' Situation Awareness in Bridge Simulations via Eye-Tracking Technology" was published in 2021. Journal: Comput Intell Neurosci.

## 1. Introduction

Improvements to pilots' situation awareness (SA) in maritime navigation are critical to reducing human errors, which have caused 75% to 96% of marine accidents over the last few years [1]. In recent years, growth in traffic densities, ship speeds, and ship sizes have led to the need to improve pilots' operational safety [2, 3]. However, current studies have focused more on evaluating operational performances, which is only a simple judgment of success or failure in cognitive results without analyzing the evolution of a pilot's SA [4]. The causation of operational errors is a deficiency of SA, which means losing the ability to hold the overall situation [5]. To evaluate unsafe behaviors in ship pilotage more effectively and practically, it is essential to investigate SA from a cognitive perspective. Before improving SA, the first problem to solve is how to accurately measure it in pilotage operations.

Some direct (questioning and/or observations) and indirect (user behaviors, physiological responses, and/or task performances) assessment methods have been proposed to measure an operator's SA based on three-level frameworks [6]. Probe-based methods are common direct measurements, such as the SA Global Assessment Technique (SAGAT) [7] and the Situation Present Assessment Method (SPAM) [8]. Nevertheless, these methods often interrupt and/or disrupt ongoing work tasks, which results in reduced task performances. Self- and observer-rating methods have also been developed to address the limitations of probe-based methods. Two frequently used rating methods are the SA Rating Technique (SART) [9] and the SA Behavioral Rating Scale (SABARS) [10]. Self-rating methods require participants to recall making rating selections at the end of an experiment, while observer-rating methods may suffer from the biases of human observers. Moreover, the eye-mind hypothesis [11] suggests that SA is highly correlated with attention [12]. Compared to direct measurements, eye-tracking technology is considered an indirect measurement that can reduce workplace interruptions and/or disruptions and may provide a more accurate and safe SA evaluation [13].

According to the literature, eye-tracking technology is focused on studies to determine the correlated relationship between an operator's cognitive state and attentional distribution through metrics such as the fixation duration, saccade count, and pupil diameter [14, 15]. This has been widely adopted in critical safety fields including aviation, medical, and nuclear power. Louw and Merat [16] demonstrated that a driver's visual attention is significantly scattered in the process of automatic driving through simulation experiments. In maritime industries, researchers have validated eye-tracking technologies in the usability of bridge layout optimal designs and bridge resource management training [17, 18]. Atik and Arslan [19] presented an assessment method using eye-tracking technology for electronic navigation competency. The results showed that eye-tracking technologies are a valuable tool to compare the significant differences between expert and novice ship officers in eight areas of interest (AOIs). With the continuous accumulation of practical experience on SA research in critical safety fields [20], eye-tracking technology is promising for future applications in ship pilotage. However, no common agreement has been made for eye-tracking metrics as correlated with SA as these have been applied in different tasks and workplaces.

The article "Correlation Evaluation of Pilots' Situation Awareness in Bridge Simulations via Eye-Tracking Technology" was published in 2021. Journal: Comput Intell Neurosci.

Fixation metrics are correlated with SA in many studies [21–23]. Several studies [24, 25] have also confirmed moderate correlations between saccade metrics and SA. Nevertheless, no study has found a significant correlation between pupil dilation or blink rate and SA [26]. It is noted that only a few studies [27] adopted multiple eye-tracking metrics, but not all had significant correlations with SA. It is generally believed that a higher SA is found when participants spend more time in a specific AOI [28]. Together, the results of the literature enable testing a general hypothesis that pilots with low and high SA levels will allocate their attention differently when exposed to the same piloting emergencies. However, the different task conditions and application purposes have not enabled a consensus on which eye-tracking metrics are correlated with SA.

The primary goal of this paper is to assess the relationships between eye movement features and SA levels. The bridge simulation experiments aim to determine a pilots' SA and obtain relevant data. Thus, this paper develops a permutation simulation approach to identify eye-tracking metrics that are significantly associated with pilots' SA levels during pilotage. The evolution processes of visual behaviors are explored in conjunction with heat maps and scan paths. The final correlation results provide a reference to develop real-time SA monitoring methods using eye movement features, which is expected to reduce piloting risks through improved pilot selection and training.

## 2. Experiments

### 2.1. Experimental Design

To assess the relationships between eye movement features and SA in ship pilotage, the designed experiment scheduled 13 exams over 3 days, each of which tested one participant who acted as a pilot in a three-person exam group. In each examination, eye-tracking technology was used to capture participant eye movement patterns, which were used to indirectly infer SA-related constructs (e.g., perception and comprehension). The SART was employed to measure SA levels before and after each exam (Figure 1) so that the pilotage tasks were not interrupted and the requirement for the continuity of eye-tracking data was maintained.

The article "Correlation Evaluation of Pilots' Situation Awareness in Bridge Simulations via Eye-Tracking Technology" was published in 2021. Journal: Comput Intell Neurosci.

When subjectively measuring SA, the nonintrusiveness and ease of implementation have made SART one of the most representative methods in self-rating techniques to measure SA levels [29]. To ensure the professionalism of questionnaires and measurement accuracy, the SART questionnaires were confirmed through safety engineering and management, maritime supervision, and senior pilot experts to adjust existing measurement items. There are three dimensions, including pilots' attentional demands, attentional supply, and situational understanding, and ten subconstructs are constructed as the measurement items in conjunction with practical pilotage situations, as listed in Table 1. The results are calculated from the formulation that SA score = understanding-(demand-supply). The SART with seven-level Likert measurement items was used to determine the pilot's SA level before and after the experiments.

The questionnaire before the experiment was recorded as SART-1. To avoid the influence of negative emotions, pressure, fatigue, and other personal factors in the experiment, SART-1 measured the subjective SA level of pilots in the memory of early pilot work. The SART-1 questionnaire in the pretest is used to predetermine the SA level in the pilotage tasks as a reference, whereas the SA level was confirmed by the SART-2 questionnaire in the posttest that was under the premise that the SA score obtained through SART-2 is the actual SA level provided that differences in the SA scores before and after the experiment are within the normal range. Otherwise, the outlier data was deleted and the corresponding pilot SART-2 score is not taken as the SA level. This was specifically designed to decrease subjective measurement errors. To facilitate the analysis, the research hypotheses divide pilots' SA into two levels based on their SART-2 score: high (above average SART-2 score) and low (below average SART-2 score). Therefore, according to the score of the SART-2, the high and low pilot SA levels were determined as the independent variables. The analysis of pupil diameter controlled the influence of external stimuli, such as light and sound, because the ship simulations were conducted indoors and completed within three consecutive days. Therefore, the pilot simulations only took differences in the pilot SA levels as the independent variable.

The article "Correlation Evaluation of Pilots' Situation Awareness in Bridge Simulations via Eye-Tracking Technology" was published in 2021. Journal: Comput Intell Neurosci.

A wearable eye-tracking device was used for correlation verification to collect the pilot's eye-tracking metrics as dependent variables, including the fixation duration, fixation counts, saccade duration, saccade counts, and pupil diameter. Visualization methods were used to study the search strategy and cognitive process of pilots in each scene, and statistical analyses were applied to identify eye movement indicators that were associated with SA levels. Heat maps and scanning paths are illustrated to visualize the pilots' eye-movement behaviors and preliminarily understand the common visual patterns of pilots and differences between the various SA groups. Although visualization techniques allow analyzing eye-tracking data in an explorative way, a statistical analysis must be performed to determine differences in attention as caused by variations in SA. Quantitatively, eye-tracking metrics are calculated for pilots in each SA group (high and low) within the piloting situation and across the AOIs. The average eye-tracking metrics among pilots with high and low SA levels were input into the permutation simulation to compare their associations.

#### 2.1.1. Participants

Pilots from different pilot stations who were enrolled in the competency qualification examination were recruited for the experiments. In the qualification examination, pilots were subjected to scenario-based comprehensive assessments, including operating skills, resilience, coordination, and psychological qualities, which were standardized by the national maritime authorities. There were 13 exams scheduled over three days; each exam tested one participant who acted as a pilot in a three-person exam group. Each pilot was a male with normal vision aged from 30 to 45 years old with a mean experience on piloting of 11.3 years and standard deviation (std.) of 1.4 years. Each pilot volunteered to participate in the experiment. All experimental procedures were approved by the maritime authority, pilot station, and school department in charge of crew training.

#### 2.1.2. Apparatus

Due to challenges in the validity and reliability of SA measurements, eye-tracking technology has become one of the major topics to investigate in the SA field. In this paper, a wireless eye-tracking device, Tobii Glasses 2 (Figure 2), was utilized to measure a pilot's gaze in real-time as they move freely in any ship pilotage setting [30]. The device consisted of four eye cameras (directed toward the subject's eyes) with a sampling rate of 100 Hz and a wide-angle full-scene camera directed toward the scene. An eye-tracking sensor and infrared light sensor were included as core components of the eye camera, which can measure the direction of eye gaze by emitting near-infrared light to the eye and receiving changes in the amount of light reflected by the cornea and sclera during eye movement.

The article "Correlation Evaluation of Pilots' Situation Awareness in Bridge Simulations via Eye-Tracking Technology" was published in 2021. Journal: Comput Intell Neurosci.

During data acquisition, the accuracy and precision of the data were used to evaluate the reliability of the wearable eye-tracking device. Accuracy is defined as the average error between the actual position of the stimulus and the position of the line-of-sight captured by the eye tracker. Precision is the extent to which the eye tracker continuously records the same fixation point, such as measured by the root mean square of a continuous sample. Based on the research aim and nature of the pilot simulation experiments, the reliability of existing eye-tracking devices can meet these requirements through reasonable configuration and calibration. Therefore, the device was set up and calibrated for each participant prior to the experiment, which was a process that required between 2 and 5 min. Moreover, the application reliability of Tobii devices has been verified in the acquisition of real-time eye-tracking data in similar driving simulations [31, 32].

#### 2.1.3. Situation Scenes

Representative situations related to pilotage tasks were selected from a database of qualification examinations, including vessel departures (scene 1), navigation in the fairway (scene 2), encounters (scene 3), poor visibility (scene 4), and anchoring (scene 5). The pilotage tasks were from the Waigaoqiao terminal phase 5 to the West Hengsha anchorage of Shanghai; the voyage plan is shown in Figure 3. The initial conditions include the type of vessel (uniformly set as the 5000TEU container ship), speed of vessel (0 knots), flood tide (1 to 2 knots), and north wind (force 3). The pilots navigated in the specific scene as emergency events successively appeared.

#### 2.1.4. AOIs

The AOIs are divided to explore the general patterns of pilots' visual attention. According to the requirements of pilots' views and good seamanship, the AOIs are divided into the electronic chart (AOI-1), outside window (AOI-2), radar (AOI-3), and maneuvering interface (AOI-4), as shown in Figure 4. The AOIs of pilots for good seamanship were confirmed by interviews with senior experts of marine technologies, including 10 from safety engineering and management, 15 from maritime supervision, and 12 senior pilot experts. They ranged from 40 to 55 years old and had an average of 15.3 (std. of 1.2) years of experience in management and pilotage. Good seamanship refers to actions taken to avoid collisions in most appropriate circumstances and conditions, which are widely recognized as the result of long-term practical experience.

The article "Correlation Evaluation of Pilots' Situation Awareness in Bridge Simulations via Eye-Tracking Technology" was published in 2021. Journal: Comput Intell Neurosci.

### 2.2. Procedure

The experiment was conducted using the SART questionnaire and eye-tracking technology received separately within two sections, which were the SA measurements and examination, respectively, as shown in Figure 5. The procedure was as follows:

1. In the measurement section, the SART questionnaires were used to obtain the pilots' SA levels before and after the pilotage experiments. The SART-1 questionnaire in the pretest was used to prejudge the real SA level.
2. In the examination section, the calibration part of the device was conducted before the experiment. The bridge simulator was then performed to sail on the preset navigation route and pass through five specific situations in turn, where the pilots conducted at least 40 min of ship pilotage tasks. During the time, the wearable wireless eye-tracking device was used to collect the pilot's gaze data.
3. Interviews for the SART-2 questionnaire were implemented to confirm the SA levels in the posttest.

## 3. Methods

### 3.1. Data Analysis

Eye-tracking features were preliminarily extracted and analyzed to identify the eye movement for different SA levels. The first step was to collect data using the eye-tracking device through the fixation counts, fixation duration, saccade counts, saccade duration, and pupil diameter. However, the temporal and spatial sampling capabilities of the eyeball limited how eye-tracking devices extract visual information from the surrounding environment. Thus, missing data at some time points were supplemented by interpolation, whereas noise was eliminated using a moving median filter. Noise refers to the data that is not marked as fixation or saccade in the raw data due to blinking or not being collected by the device. Taking the gaze data in a fragment, for example, indicates that the noise was effectively removed after filtering the gaze data, as shown in Figure 6.

Subsequently, there are two complementary ways to identify and calculate the fixation or saccade features of signals. Due to the rapidly declining fixation accuracy when the sightline was moved out of the central field of vision, the velocity-threshold identification (I-VT) was adopted to classify eye-tracking types (i.e., fixation and saccade) [33]. The I-VT extracts gaze data with frequencies <3 Hz and fixation times of 50–600 ms while defining the threshold set to an eye movement speed of 30°/s. Samples above the threshold are saccade, while those below the threshold are fixation. Moreover, the coordinate positions of the fixation samples were recorded in conjunction with the pilot's view. In feature identification, the gaze position relative to the pilots' visual view is another important way to acquire feature types, including fixation and saccade.

The article "Correlation Evaluation of Pilots' Situation Awareness in Bridge Simulations via Eye-Tracking Technology" was published in 2021. Journal: Comput Intell Neurosci.

Visual behaviors were identified by registered coordinates using the eye-tracking device (coordinates of the fixation are smooth and the saccades are undulating). The gaze data along with the marked position allows determining the fixation duration, fixation count, saccade duration, and saccade count, as seen in Figure 6. The minimum acquisition parameter for the pupil diameter using the eye-tracking device was set to 2 mm by default. Linear interpolation was used due to the lower loss and extreme values in the raw data; the processed data is shown in Figure 7 [34]. In general, the output types of the eye-tracking devices combined with identification and calculation methods allow the signal features to be divided into fixation, saccade, and noise. Noise accounts for 16.8% (87.6 min) of the total experimental duration and is within the expected range.

### 3.2. Permutation Simulations

To evaluate the correlation, the data were analyzed statistically, including parametric tests (*t*-test), nonparametric tests (Mann–Whitney *U* test), and permutation simulations. Parametric tests are effective for good sample conditions (approximately normal), but the eye-movement data did not meet the distribution requirements [35]. Furthermore, as the permutation simulations resample the data to construct empirical distributions rather than ranking them using nonparametric tests, the simulations had a higher statistical power than other nonparametric techniques [36]. Therefore, the statistical analysis included a permutation to evaluate the eye-tracking data of the AOIs in corresponding pilotage scenes. The basic concept of the permutation simulations is to perform all possible permutations for given eye-tracking data and generate the reference distribution of the test statistics by resampling the data and recalculating the statistics to determine the *p*-value of the test. With permutations, the calculated *t*-value was used as a measure of the group's difference, which was tested against an empirical sampling distribution. It was then determined whether the new *t*-value was extreme or smaller than the observed value. If a *t*-value greater than the observed value is produced at the 10,000 resampling, the probability of such an extreme outcome is only about 1/10,000. It is noted that the *t*-value is used to measure the differences between groups and is not a statistic to compare with the parameter *t* distribution. This study considered a 95% confidence level (*p* < 0.05) as significant and a 90% confidence level (*p* < 0.1) as moderately significant.

The article "Correlation Evaluation of Pilots' Situation Awareness in Bridge Simulations via Eye-Tracking Technology" was published in 2021. Journal: Comput Intell Neurosci.

## 4. Results

To validate the research hypotheses, the SART scores before and after the experiment were gathered without abnormal change. The pilots were divided into a high SA group of seven participants (mean = 24.5, standard deviation = 5.13) and a low SA group of six participants (mean = 15.2, standard deviation = 4.37) based on the SART-2 score (mean = 20.13, standard deviation = 5.83) after the experiments. Although this classification method is not sophisticated, the subjectivity of the SART technique can be reduced by conducting questionnaires before and after the experiments and segregating based on average scores.

### 4.1. Visualization

To avoid confusing the effects of AOIs on the differences in the pilots' SA levels and eye-tracking metrics, the AOIs were selected individually for visualized analysis. The first step allows researchers to extract eye movement features using the eye-tracking device, and the corresponding coordinates and pilot's view were recorded synchronously. Taking the gaze data during departure (scene 1) as an example, the discrete degree in the high SA group was greater than that in the low SA group, indicating pilots in the high group may scan more areas (Figure 8). Thus, the relatively static fixation segment with a certain time continuity is defined as the “background” subview, and colors ranging from green to red were used to represent how much an individual (or group) attended different AOIs in a scene based on the heat map. Additionally, the scan paths show the visual search strategy of an individual (or group). Therefore, it is possible to analyze the observed information of the AOIs by selecting unified views (mapping backgrounds of the heat map and scan path) to summarize the eye movement features under different subviews. The visualization outputs and analyses of these recorded eye movements help interpret the results qualitatively to better understand the quantitative results.

To visually compare the attentional allocation and scanning strategies of different individuals in the two SA groups, the pilot's visual behaviors are illustrated using heat maps and scan paths from the eye-tracking metrics in the five scenes of the examination. Scene 1 and scene 3 were selected as examples for the visualization results. The heat map analysis results demonstrate two things: pilots mainly focus on the electrical chart (AOI-1) and outside window (AOI-2) in ship pilotage, and the fixation duration of AOI-1 or AOI-2 in the two SA groups differ from the visual area and color of the map, as shown in Figure 9. Pilots in the high and low SA groups paid more attention to AOI-2 and AOI-1, respectively. These results are also reflected in the heat maps of the other three scenes (data not shown). This suggests that selective attentional distributions between the two AOIs may be correlated with participants' SA level.

The article "Correlation Evaluation of Pilots' Situation Awareness in Bridge Simulations via Eye-Tracking Technology" was published in 2021. Journal: Comput Intell Neurosci.

The scan path is the presentation of the order and position of fixation points on the AOIs, in which the dot indicates the fixation duration, and the number represents the order of fixation points. The results of the scan path analysis show that participants mainly scan back and forth in AOI-2. Moreover, the saccade frequency is selected as a preliminary analysis of the pilot's saccade pattern, which is defined as the saccade count per unit time of the pilots between AOI-1 and AOI-2. A further finding is that the saccade frequency in the high SA group was higher than that in the low SA group, indicating there are differences between the scanning paths of the two AOIs back and forth, as shown in Figure 10. This is because pilots in the high SA group frequently confirm the perceptual elements in the situations for scene 1 and scene 3. Thus, there were timely updates to the mental model to make accurate behavioral predictions. These results are reflected in the scan paths of the other three scenes (data not shown). Together, the present findings confirm that the scanning strategies may be associated with the SA level in ship pilotage.

### 4.2. AOI Analysis

The mean fixation duration (i.e., the average of fixation duration as a percentage of the duration of the corresponding scene) and mean saccade counts (i.e., the average counts of saccades per second for the corresponding scene of pilots) were selected as statistical indicators for preliminary quantitative analyses, which respectively imply the attention of individuals for AOIs and the complexity of obtaining information. In actual ship pilotage, differences in pilot skills cause various completion times of the pilotage tasks in corresponding scenes. Thus, the mean fixation duration is expressed as a percent. The error bars in Figure 11 show the standard deviation of the sample mean.

The mean fixation durations of AOI-1 and AOI-2 are compared to verify the differences of the fixations for the two SA groups, as shown in Figures 11(a) and 12(b). As the total fixation durations of AOI-3 and AOI-4 across all scenes account for less than 5% of the task duration, they are not statistically different. Hence, only AOI-1 and AOI-2 were statistically analyzed. The mean fixation duration of AOI-1 across all scenes in the high SA group accounts for 75.4% of the total effective fixation duration, while that of AOI-2 across all scenes in the low SA group accounts for 62.3% of the total effective fixation duration. In real-world pilotage, this can be explained from two aspects: ship pilotage is a team task, where crucial information of the radar (AOI-3) and maneuvering interface (AOI-4) is mainly obtained in the form of communications with the captain and helmsman to retell maneuvering commands. As the data for AOI-3 and AOI-4 can be displayed in AOI-1 through the information integration function, it is easier for AOI-1 to occupy the attentional resources from AOI-3 and AOI-4. Additionally, the mean saccade count, total mean saccade count within AOI-1 across all scenes (73.794 c/s), and the total mean saccade count within AOI-2 across all scenes (75.114 c/s) of the low SA group are greater than those of the high SA group (mean saccade count of 39.203 c/s within AOI-1 across all scenes and of 58.339 c/s within AOI-2 across all scenes), as seen in Figures 11(c) and 11(d). This indicates that pilots in the low SA group have a relatively poor ability to obtain information, and the specific visual behavior is manifest as repeated scanning in specified AOIs. These saccade behaviors are specifically shown in the scan path of the low SA group, which are performed primarily in AOI-1 (Figure 10(d)).

The article "Correlation Evaluation of Pilots' Situation Awareness in Bridge Simulations via Eye-Tracking Technology" was published in 2021. Journal: Comput Intell Neurosci.

To analyze different scenes, the mean fixation duration of AOI-2 for the high SA group during the encounter (scene-3) was the longest (0.370, std. = 0.124), and anchoring (scene-5) was the least (0.143, std. = 0.051), as seen in Figure 11(b). This result is in line with reality:

1. Good seamanship in scene 3 tends to combine experience with behavior predictions, which is necessary to anticipate the development of relative courses and distances between ships in AOI-2 in real time.
2. In scene 5, the visual behaviors in the AOI-1, which should be considered to obtain information elements including the ship position, depth, and anchorage-prohibited areas, occupy most of the attention resources from AOI-2.

The total mean saccade count at AOI-2 for pilots in the high and low SA groups during the encounter (scene 3) (38.701 c/s) and poor visibility (scene 4) (35.435 c/s) are higher than those in other scenes (13.167 c/s of scene 1, 24.710 c/s of scene 2, and 21.441 c/s of scene 5). This indicates that pilots have higher perceptual requirements in the complex environments of scene 3 and scene 4 (Figure 11(d)). During anchoring (scene 5), the mean saccade count of the low SA group in AOI-1 is the highest (20.644 c/s and std. = 3.87), which implies that the main perceptual information acquisition may come from AOI-1 and pilots in the low SA group were not familiar with its contents (Figure 11(c)).

The article "Correlation Evaluation of Pilots' Situation Awareness in Bridge Simulations via Eye-Tracking Technology" was published in 2021. Journal: Comput Intell Neurosci.

### 4.3. Correlation Evaluation

To determine whether these differences are statistically significant, averages of the eye-tracking metrics from each SA group are compared across the AOIs using the permutation simulation technique. As before, AOI-1 and AOI-2 are selected for statistical analysis as they are the objects of primary fixation and saccades in the visualized and AOI analyses. The statistical differences between the eye-tracking metrics and SA levels in the two AOIs across the five scenes are calculated in the permutation simulations. Thus, descriptive statistics of the five eye-movement metrics (fixation count, fixation duration, saccade count, saccade duration, and pupil diameter) for the two SA groups and the results of the statistical tests are summarized in Tables 2 and 3.

In the statistical analysis of AOI-1, the test results show that the fixation count is significantly correlated with the SA level across four scenes (scene 1 at *p* = 0.043 < 0.05, scene 2 at *p* = 0.035 < 0.05, scene 3 at *p* = 0.034 < 0.05, and scene 4 at *p* = 0.024 < 0.05). The fixation duration is significant across three scenes (scene 2 at *p* = 0.034 < 0.05, scene 3 at *p* = 0.043 < 0.05, and scene 4 at *p* = 0.036 < 0.05), as listed in Table 2. In scene 5, the pilot's SA level impacts the fixation duration (*p* = 0.092 < 0.1). These outcomes demonstrate that the high SA pilots may be inclined to take more fixation behaviors toward ship navigation and environmental information from AOI-1 across scene 2, scene 3, and scene 4. Specifically in scene 3, as the encounter situation changes in real time, the pilots are required to scan the scene to obtain any necessary feedforward information related to ship collision hazards and take safe pilotage measures without neglecting stored materials. The descriptive statistics related to scene 3 show that pilots with a lower SA have a higher mean on all fixation metrics than those in other scenes. This demonstrates that they urgently need to obtain more feedforward information in real time (Table 2).

As the saccade behaviors reflect how easy it is for pilots to obtain information in a specified AOI, the statistical tests show that two saccade metrics are moderately significantly associated with the SA level, indicating that high SA pilots can obtain the necessary information from AOI-1 in corresponding scenes. These are the saccade count (*p*_scene-3_ = 0.086 < 0.1, *p*_scene-4_ = 0.075 < 0.1, and *p*_scene-5_ = 0.087 < 0.1) and saccade duration (*p*_scene-1_ = 0.079 < 0.1). In scene 4, the saccade duration (*p* = 0.05 ≤ 0.05) may be more conducive to distinguish this ability between pilots with different SA levels. These results show that the pilot SA level influences saccade behaviors on AOI-1 across scene 1, scene 3, scene 4, and scene 5. For the descriptive statistics related to scene 4, the poor visibility is not conducive for pilots to obtain real-time environmental information by scanning the scene. Thus, pilots with high SA levels have a higher mean on all fixation metrics and a lower mean on all saccade metrics than in the other scenes. This demonstrates that they are limited by environmental conditions and can only acquire pilot-related information through effective fixation behaviors in AOI-1. The high SA has a better ability to understand the necessary feedforward information in AOI-1, while saccade behaviors are the least (Table 2).

The article "Correlation Evaluation of Pilots' Situation Awareness in Bridge Simulations via Eye-Tracking Technology" was published in 2021. Journal: Comput Intell Neurosci.

The test results for the analysis of AOI-2 show that the fixation count is significantly correlated with the SA level across four scenes (scene 1 at *p* = 0.038 < 0.05, scene 2 at *p* = 0.027 < 0.05, scene 3 at *p* = 0.032 < 0.05, and scene 4 at *p* = 0.034 < 0.05), and the fixation duration across three scenes (scene 2 at *p* = 0.033 < 0.05, scene 3 at *p* = 0.014 < 0.05, and scene 4 at *p* = 0.047 < 0.05), as listed in Table 3. In scene 5, the pilot's SA level also impacts the fixation count at *p* = 0.086 < 0.1. These outcomes demonstrate that high-SA pilots tend to adopt more fixation behaviors toward real-time environmental information from AOI-2 across scene 2, scene 3, and scene 4. Specifically in scene 3, pilots with high SA levels were inclined to obtain feedforward information that was sufficient to predict situations in near future through AOI-2, and then effective predictions were made based on their experience and knowledge. The descriptive statistics related to scene 3 show that pilots with higher SAs have a greater mean for all fixation metrics than those in other scenes, indicating they are good at piloting based on empirical perception and can reduce their overdependence on navigation equipment (Table 3).

The significant statistical differences between the saccade duration and SA level in AOI-2 are verified in scene 1 and scene 4 (*p*_scene 1_ = 0.040 < 0.05 and *p*_scene 4_ = 0.042 < 0.05), as listed in Table 3. In scene 2 and scene 3, the pilot's SA level impacts the two saccade metrics: saccade count (*p*_scene 3_ = 0.054 < 0.1) and saccade duration (*p*_scene 2_ = 0.098 < 0.1 and *p*_scene 3_ = 0.075 < 0.1). These results show that only in scene 3 do the pilots' two saccade metrics correlate with the SA level. In scene 3, pilots have a higher mean on all saccade metrics than in the other scenes, indicating they are needed to comprehensively understand and master environmental information from AOI-2 through saccade behaviors to accurately prejudge ship encounter situations in the near future (Table 3), whereas the pupil diameter is not significant for AOI-1 and AOI-2 across all scenes due to the possibility of individual differences, as listed in Tables 2 and 3. Combined with the correlation evaluation of AOI-1 and AOI-2 in the five scenes, these results provide the possibility for future studies to identify pilots' SA levels in different scenes using fixation and saccade metrics.

The article "Correlation Evaluation of Pilots' Situation Awareness in Bridge Simulations via Eye-Tracking Technology" was published in 2021. Journal: Comput Intell Neurosci.

The correlation analysis identifies different significant eye-tracking metrics from AOI-1 and AOI-2 in each pilotage scene, as shown in Figure 12. The correlation in AOI-1 indicates that the pilots' SA level affects the eye movement metrics for AOI-1 across the corresponding scene, and the correlation in AOI-2 is defined accordingly. Correlative metrics are adopted to realize the recognition of statistical differences throughout the scenes, which should be owned by both AOIs and be above the average (more than two of five) in one scene. Thus, scenes that satisfy the above condition are defined as the corresponding scene that can effectively reflect a pilot's SA level through correlated eye-tracking metrics, which combines the correlation results of AOI-1 and AOI-2. A pilot's high SA level implies his or her ability to complete pilotage tasks independently and excellently, and the eye-tracking metrics are found to be correlated with the SA level. Therefore, subsequent studies are expected to effectively reflect the SA level of pilots in ship pilotage through associated eye-tracking metrics.

In summary, the fixation count, fixation duration, and saccade count are related to the SA level in scene 3 and the fixation count, fixation duration, and saccade duration are determined in scene 4. Conversely, scene 1, scene 2, and scene 5 tended to show pilots adopting negative fixation behaviors due to the possible development of cognitive states, such as adaptive transition in the preexperiment and relaxation or fatigue caused by simple and long-term tasks. These negative behaviors include adopting negative coping modes due to the external environment or his/her own emotions, which are manifested as visual behaviors inconsistent with the reality of ship pilotage. This indicates that the pilot SA level cannot be effectively characterized by eye-tracking metrics in such scenes based on the current research results. To effectively monitor the evolution of the pilot's SA cognitive states through physiological indicators in scene 1, scene 2, and scene 5, multiple indicators are needed for further consideration, such as heart rate variability (HRV) [37], electrodermal activity (EDA) [38], electromyography (EMG) [39], and electroencephalogram (EEG) [40].

The article "Correlation Evaluation of Pilots' Situation Awareness in Bridge Simulations via Eye-Tracking Technology" was published in 2021. Journal: Comput Intell Neurosci.

## 5. Discussion

The AOIs account for at least 90% of the 13 pilots' visual areas, where AOI-3 and AOI-4 together occupy less than 5% of the simulation experiment duration. The pilots' visual features (fixation, saccade, and coordinates) were extracted using eye-tracking technology to calculate the proportion of the cumulative time for these visual behaviors in the AOIs to the total effective time. The mean saccade counts in the low SA group for AOI-1 and AOI-2 are both higher than the high SA group. However, the mean fixation duration of the low SA group is higher than the high SA group for AOI-1, whereas the high SA group exceeds the low SA group for AOI-2. This is because the high SA group members with more practical experience tend to observe and analyze scenes through AOI-2 rather than relying on equipment such as electronic charts (AOI-1). In general, the heat map and saccade paths for the pilots' visual behaviors intuitively confirm the conventional understanding of piloting experience that high SA pilots are inclined to observe the environment from a real perspective rather than through equipment as is true for low SA pilots.

Permutation simulations were conducted on the gaze data for the pilots in both SA groups. In the five scenes, the eye-tracking metrics for AOI-1 are most associated with the SA in scene 2, scene 3, and scene 4, while the visual behaviors for AOI-2 are confirmed in scene 3 and scene 4. The correlation analysis of the eye-tracking features in each scene identifies the fixation count, fixation duration, and saccade count as eye-tracking metrics associated with pilots' SA levels in scene 3. The fixation count, fixation duration, and saccade duration are identified in scene 4. The findings for the fixation metrics agree with reports in previous studies [27, 41]. Moreover, there was no significant correlation found between the pupil dilation and SA, which is similar to previous studies [26]. However, distinct from previous reports [42], these results demonstrate the significant correlation of the saccade metrics with SA. Comparing these results with other studies indicates that this study systematically and comprehensively explores the relationship between eye movement features and SA for ship pilots. Further, to monitor pilots' cognitive competency through physiological indicators over the entire piloting process, scene 3 and scene 4 are identified as those with correlations between the SA level and eye-tracking metrics. Thus, there is a possibility that a pilot's SA level can be effectively characterized using eye-tracking metrics in such scenes. In follow up on studies, these findings will lay a foundation to construct the overall monitoring framework.

The article "Correlation Evaluation of Pilots' Situation Awareness in Bridge Simulations via Eye-Tracking Technology" was published in 2021. Journal: Comput Intell Neurosci.

For correlation verification, the relationship between pilots' eye-tracking metrics and their SA level is associated with the AOIs for the different scenes. This study shows that ship pilotage in encounters (scene 3) and poor visibility (scene 4) are more likely to increase visual behaviors, including fixation and saccades, in AOI-1 and AOI-2. However, the permutation results are inconsistent with the preliminary statistics, such as the difference in the mean fixation duration of the SA groups for AOI-1 during departure (scene 1), which has not been verified. Therefore, the main limitation of this study is the sample size of ship pilots. As the ship pilotage process is complete and standardized, and dynamic simulation scenes need to be realized based on large ship maneuvering simulators, the number of potential participants is limited. To compensate for the small sample size, statistical methods in this study increase the capability of analysis through resampling (10,000 samples) and recalculating data statistics, but the applicability of the results is inevitably affected.

The performance issue of eye-tracking devices is also a limitation. When a pilot acts quickly, the data may not be collected because the acquisition speed of the eye-tracking device cannot keep up, which causes reduced local data. Although interpolation helps supplement the data, it inevitably affects the significance level of the correlation results. Another limitation is the lack of integration with other physiological measures. The SA level is not only correlated with eye movement features but is also related to other physiological measurement metrics, as confirmed in previous studies [43–45]. Therefore, combining multiple physiological metrics to investigate their correlation with the SA level is a basic research direction in SA assessments.

## 6. Conclusion

Pilots' SA is associated with pilotage safety in maritime navigation. In the case of emergencies, pilots are required to control the situation. The SA is a specific representation of the cognitive state and the essence of pilots' behaviors, which includes the cognitive processes of perception, understanding, and prediction. Although unsafe behaviors are regarded as a direct causation of pilotage accidents, the essential role of cognitive mechanisms in maritime pilot behaviors is not fully understood in the current field of safe pilotage. The application of monitoring technologies for pilots' cognitive competency is the key issue. This study evaluates the utility of eye-tracking technologies and analyzes the correlation of eye-tracking metrics with SA levels to determine whether such metrics can effectively differentiate ship pilots with high and low SA levels in a specific pilotage scene. Qualitative results (presented as scan paths and heat maps) for the pilots' SA in a bridge simulator test reveal that pilots in the high SA group focused on the AOI-2 (outside window), whereas the low SA group members focused on AOI-1 (electronic chart). Furthermore, quantitative analyses via permutation simulations determined that different eye-tracking metrics are associated with the SA level in the different scenes. These results demonstrate the availability of eye-tracking technologies in poor visibility and encounter subscenes, which provides the opportunity for the subsequent applications of cognitive ergonomics in improved pilotage safety.

The article "Correlation Evaluation of Pilots' Situation Awareness in Bridge Simulations via Eye-Tracking Technology" was published in 2021. Journal: Comput Intell Neurosci.

Understanding the pilots' attention allocation pattern as recognized by eye-tracking technology can objectively distinguish the SA level and realize the accurate and rapid detection of at-risk cognitive states to provide an important reference for personnel preliminary screening. Moreover, the outcomes of this study contribute to the subsequent construction of pilots' SA recognition models based on correlation verifications of eye-tracking metrics. This is conducive to the optimal allocation of training resources and targeted improvements to visual behaviors. Therefore, this study yields not only immediate benefits in connecting eye-tracking metrics to pilots' attentional allocation and SA but also the long-term benefits in opening new avenues to monitor cognitive statuses and preventing unsafe behaviors.

## Figures and Tables

**Figure 1:** Experimental framework of the maritime pilotage simulations.

**Figure 2:** Tobii Glasses 2 (photo courtesy of Tobii).

**Figure 3:** Voyage plan with various scenes in the ship pilotage simulations.

**Figure 4:** AOIs in the ship pilotage simulations.

**Figure 5:** Experimental procedure to determine SA levels in pilotage tasks.

**Figure 6:** Fragment of the processed fixation position measurements.

**Figure 7:** Fragment of the processed pupil diameter measurements.

**Figure 8:** Gaze data of SA groups in the departure (scene 1).

**Figure 9:** Heat map of departure (scene 1) and encounter (scene 3). (a) Heat map of high SA group in scene 1. (b) Heat map of low SA group in scene 1. (c) Heat map of high SA group in scene 3. (d) Heat map of low SA group in scene 3.

**Figure 10:** Scan path of departure (scene 1) and encounter (scene 3). (a) Scan path of high SA group in scene 1. (b) Scan path of low SA group in scene 1. (c) Scan path of high SA group in scene-3. (d) Scan path of low SA group in scene-3.

The article "Correlation Evaluation of Pilots' Situation Awareness in Bridge Simulations via Eye-Tracking Technology" was published in 2021. Journal: Comput Intell Neurosci.

**Figure 11:** Mean duration and saccades in all scenes. (a) Mean fixation duration in AOI-1. (b) Mean fixation duration in AOI-2. (c) Mean saccade count in AOI-1. (d) Mean saccade count in AOI-2.

**Figure 12:** Correlation between eye-tracking metrics and SA in all scenes.

**Table 1:** SART measurement dimensions.

Dimension	Construct	Measurement item
Attentional demands	Instability of situation	Stability of traffic environment and vessel in the pilotage (without emergency)
	Variability of situation	Number of variables, including navigational and environmental elements, that should be the focus in pilotage
	Complexity of situation	Complexity of the traffic in pilotage waters

Attentional supply	Arousal	Alertness of pilots in pilotage
	Spare mental capacity	How much residual energy should be used to handle emergencies in pilotage
	Concentration	Degree of concentration at initial pilotage
	Division of attention	Ability to notice multiple information variables simultaneously in pilotage

Understanding of the situation	Information quantity	Amount of information received and understood
	Information quality	Reliability of perceived information
	Familiarity	Familiarity of pilotage waters

**Table 2:** Eye-tracking metrics acquired for AOI-1 in all scenes.

AOI-1	Eye-tracking metrics	High SA		Low SA		Permutation results	
		Mean	Std.	Mean	Std.	Welch's *t*	*p*-value
Scene 1	**Fixation count**	8.835	1.127	15.571	1.235	2.413	**0.043** ^**b**^
	Fixation duration	14.327	1.614	21.366	2.386	0.463	0.626
	Saccade count	4.946	4.089	11.306	1.370	1.484	0.164
	**Saccade duration**	0.704	0.338	0.716	0.303	2.145	**0.079** ^**a**^
	Pupil diameter	4.437	0.860	4.329	1.179	1.574	0.425

Scene 2	**Fixation count**	14.044	3.485	23.354	2.437	2.675	**0.035** ^**b**^
	**Fixation duration**	16.649	3.939	23.124	1.425	2.687	**0.034** ^**b**^
	Saccade count	6.913	4.382	13.212	1.549	1.054	0.266
	Saccade duration	0.512	0.168	0.559	0.090	1.375	0.339
	Pupil diameter	3.899	0.633	4.422	1.107	0.537	0.704

Scene 3	**Fixation count**	16.239	4.466	23.905	2.936	2.363	**0.034** ^**b**^
	**Fixation duration**	23.726	1.976	27.961	2.436	2.075	**0.043** ^**b**^
	**Saccade count**	6.964	3.399	14.445	3.816	1.934	**0.086** ^**a**^
	Saccade duration	0.471	0.297	0.826	0.434	1.454	0.347
	Pupil diameter	4.435	0.756	4.591	1.124	0.865	0.697

Scene 4	**Fixation count**	19.096	1.063	15.042	2.171	2.776	**0.024** ^**b**^
	**Fixation duration**	26.28	2.915	19.595	3.456	2.462	**0.036** ^**b**^
	**Saccade count**	0.445	0.323	0.674	0.334	1.817	**0.075** ^**a**^
	**Saccade duration**	0.449	0.322	0.674	0.332	2.475	**0.050** ^**b**^
	Pupil diameter	4.214	0.775	4.356	1.096	−0.183	0.849

Scene 5	Fixation count	6.922	2.775	16.993	1.654	1.078	0.237
	**Fixation duration**	5.314	1.282	11.416	1.844	1.873	**0.092** ^**a**^
	**Saccade count**	4.846	4.19	12.082	2.677	1.923	**0.087** ^**a**^
	Saccade duration	0.646	0.291	0.726	0.258	1.621	0.343
	Pupil diameter	4.035	0.748	4.221	1.143	0.964	0.694

^a^ *p*<0.1, ^b^*p* < 0.05.

The article "Correlation Evaluation of Pilots' Situation Awareness in Bridge Simulations via Eye-Tracking Technology" was published in 2021. Journal: Comput Intell Neurosci.

**Table 3:** Eye-tracking metrics acquired for AOI-2 in all scenes.

AOI-2	Eye-tracking metrics	High SA		Low SA		Permutation results	
		Mean	Std.	Mean	Std.	Welch's *t*	*p*-value
Scene 1	**Fixation count**	18.465	6.694	6.378	2.875	2.236	**0.038** ^**b**^
	Fixation duration	17.318	7.874	4.299	1.806	0.531	0.677
	Saccade count	9.489	5.121	11.241	2.447	0.751	0.526
	**Saccade duration**	0.546	0.306	0.808	0.188	2.214	**0.040** ^**b**^
	Pupil diameter	4.324	0.867	4.391	1.276	-0.161	0.888

Scene 2	**Fixation count**	14.226	2.986	4.776	2.971	2.486	**0.027** ^**b**^
	**Fixation duration**	13.066	5.919	2.984	2.044	2.195	**0.033** ^**b**^
	Saccade count	9.974	4.894	10.510	1.050	1.452	0.293
	**Saccade duration**	0.559	0.274	0.687	0.044	1.746	**0.098** ^**a**^
	Pupil diameter	3.876	0.576	4.171	1.177	0.715	0.537

Scene 3	**Fixation count**	24.943	4.373	15.664	1.943	2.263	**0.032** ^**b**^
	**Fixation duration**	25.599	6.601	14.867	4.013	2.353	**0.014** ^**b**^
	**Saccade count**	17.186	8.003	15.891	1.904	1.856	**0.054** ^**a**^
	**Saccade duration**	0.895	0.336	0.889	0.083	1.782	**0.075** ^**a**^
	Pupil diameter	4.369	0.843	4.556	1.189	0.382	0.692

Scene 4	**Fixation count**	19.911	7.567	5.282	3.674	2.337	**0.034** ^**b**^
	**Fixation duration**	17.563	10.156	3.476	2.899	2.149	**0.047** ^**b**^
	Saccade count	13.404	8.256	14.216	1.606	1.996	0.390
	**Saccade duration**	0.724	0.339	0.723	0.315	2.353	**0.042** ^**b**^
	Pupil diameter	4.214	0.826	4.348	1.144	-0.306	0.803

Scene 5	**Fixation count**	15.202	3.116	5.566	2.426	1.626	**0.086** ^**a**^
	Fixation duration	15.654	4.739	7.893	2.454	1.221	0.298
	Saccade count	10.141	5.284	11.214	2.589	1.369	0.236
	Saccade duration	0.769	0.284	0.684	0.244	1.294	0.396
	Pupil diameter	3.934	0.737	4.222	1.073	0.425	0.618

^a^ *p*<0.1, ^b^*p* < 0.05.

## Data Availability

All data generated or used during the study can be obtained from the experimental protocol in the submitted article.
